The article "Development and Validation of a Novel Clinical Prediction Model to Predict the Risk of Lung Metastasis from Ewing Sarcoma for Medical Human-Computer Interface" was published in 2022. Journal: Comput Intell Neurosci.

# Development and Validation of a Novel Clinical Prediction Model to Predict the Risk of Lung Metastasis from Ewing Sarcoma for Medical Human-Computer Interface

**DOI:** 10.1155/2022/1888586

**Published:** 2022-03-29

**Authors:** Wenle Li, Tao Hong, Chan Xu, Bing Wang, Zhaohui Hu, Qiang Liu, Haosheng Wang, Shengtao Dong, Wei Kang, Chengliang Yin

**Affiliations:** ^1^Department of Orthopedics, Xianyang Central Hospital, Xianyang, China; ^2^Clinical Medical Research Center, Xianyang Central Hospital, Xianyang, China; ^3^Department of Cardiac Surgery, Fuwai Hospital Chinese Academy of Medical Sciences, Shenzhen, China; ^4^Department of Spine Surgery, Liuzhou People's Hospital, Liuzhou, China; ^5^Department of Orthopaedics, The Second Hospital of Jilin University, Changchun, China; ^6^Department of Spine Surgery, Second Affiliated Hospital of Dalian Medical University, Dalian, China; ^7^Department of Mathematics, Physics and Interdisciplinary Studies, Guangzhou Laboratory (Bioland Laborarory, Guangzhou Regenerative Medicine and Health Guangdong Laboratory), Guangzhou 510005, Guangdong, China; ^8^Faculty of Medicine, Macau University of Science and Technology, Macau, China

## Abstract

**Background:**

This study aimed at establishing and validating a quantitative and visual prognosis model of Ewing Sarcoma (E.S.) via a nomogram. This model was developed to predict the risk of lung metastasis (L.M.) in patients with E.S. to provide a practical tool and help in clinical diagnosis and treatment.

**Methods:**

Data of all patients diagnosed with Ewing sarcoma between 2010 and 2016 were retrospectively retrieved from the Surveillance, Epidemiology, and End Results (SEER) database. A training dataset from the enrolled cohorts was built (*n* = 929). Predictive factors for L.M. were identified based on the results of multivariable logistic regression analyses. A nomogram model and a web calculator were constructed based on those key predictors. A multicenter dataset from four medical institutions was established for model validation (*n* = 51). The predictive ability of the nomogram model was evaluated by the receiver operating characteristic (ROC) curve and calibration plot. Decision curve analysis (DCA) was applied to explain the accuracy of the nomogram model in clinical practice.

**Results:**

Five independent factors, including survival time, surgery, tumor (*T*) stage, node (N) stage, and bone metastasis, were identified to develop a nomogram model. Internal and external validation indicated significant predictive discrimination: the area under the ROC curve (AUC) value was 0.769 (95% CI: 0.740 to 0.795) in the training cohort and 0.841 (95% CI: 0.712 to 0.929) in the validation cohort, respectively. Calibration plots and DCA presented excellent performance of the nomogram model with great clinical utility.

The article "Development and Validation of a Novel Clinical Prediction Model to Predict the Risk of Lung Metastasis from Ewing Sarcoma for Medical Human-Computer Interface" was published in 2022. Journal: Comput Intell Neurosci.

**Conclusions:**

In this study, a nomogram model was constructed and validated to predict L.M. in patients with E.S. for medical human-computer interface—a web calculator (https://drliwenle.shinyapps.io/LMESapp/). This practical tool could help clinicians make better decisions to provide precision prognosis and treatment for patients with E.S.

## 1. Introduction

Ewing sarcoma (E.S.) is the second most frequent primary malignant tumor among children and adolescents, especially in the age group of 4 to 15 years; it was first reported by James Ewing in 1921 [1–4]. E.S. is usually caused by a chimeric fusion oncogene; the most common one (80–85%) is t (11; 22) (q24; q12) [5, 6]. As a result, the multimodal therapeutic approaches involving a combination of chemotherapy, surgery, and radiotherapy for local control were applied for several decades. Overall survival (O.S.) of E.S. increased gradually from about 10% to 55–75% within five years [3, 7–10]. E.S. is identified as an aggressive tumor based on its clinical performance, characterized by rapid growth, high risk of metastases [2, 11], and poor prognosis [3]. The 5-year O.S. of E.S. patients is below 30% [4, 9], while about 25%–35% undergo metastasis [3, 12, 13]. The lung is the most vulnerable site for metastasis [2, 4]. Patients with isolated L.M. showed a slight improvement [3, 4]. However, the 5-year event-free survival (EFS) remains dismal at 42%.

Previous research mainly focused on potential risk factors for prognosis and metastasis [2, 13–23], while few studies integrated multiple independent factors to predict L.M. Thus, it is imperative to accurately predict the probability of L.M. As a prediction tool, the nomogram possess advantages of visualization, quantification, and accuracy, which is widely used to assess tumor prognosis and metastasis [5, 24–31].

Although E.S. was much more common in the white population, the morbidity of E.S. in the U.S. was 2.93 per 1,000,000 [32]. Limited by the incidence, our study cohort was extracted from the Surveillance, Epidemiology, and End Results (SEER) database, which consists of 18 cancer registries covering approximately 30% of the total U.S. population.

The purpose of this study was to establish a nomogram model based on the SEER database and externally validate it by a dataset from four medical institutions. Subsequently, a medical human-computer interface (web calculator) was designed to efficiently and accurately evaluate the risk for various E.S. patients via Internet [33]. This model could provide clinicians with quantitative information to make fast and scientific decisions and better clinical planning, for delivering precision healthcare to patients.

The article "Development and Validation of a Novel Clinical Prediction Model to Predict the Risk of Lung Metastasis from Ewing Sarcoma for Medical Human-Computer Interface" was published in 2022. Journal: Comput Intell Neurosci.

## 2. Materials and Methods

The SEER database is publicly available, and the patients are anonymous. Hence, the informed consent of patients was not required for this study [21, 34].

### 2.1. Patients and Data Collection

This retrospective study extracted data of E.S. patients who were diagnosed and treated between 2010 and 2016 from the SEER database as the training cohort by using SEER*∗*STAT (8.3.5) software.

The inclusion criteria were as follows: (1) diagnosis of E.S. with ICD-O-3/WHO 2008 morphology code 60 and (2) complete clinical information. The exclusion criteria were as follows: (1) information on clinicopathological and survival time was missing or unavailable and (2) cases with other primary tumor diseases and unknown metastatic status.

The demographic and clinical variables of age, race, survival time, primary site, laterality, *T* stage, N stage, surgery, radiation, chemotherapy, and distant metastasis were recorded from the SEER database using SEER*∗*STAT (8.3.5) software.

Four medical institutions, including the Second Affiliated Hospital of Jilin University, the Second Affiliated Hospital of Dalian Medical University, Liuzhou People's Hospital, and Xianyang Central Hospital, provided external validation. There were three investigators responsible for the acquisition and processing of data in each institution for the external validation. Two of them extracted data, and a third investigator conducted the accuracy checks. All data have been checked for consistency and sorted by date using Microsoft Excel (Microsoft Excel, 2013, Microsoft, Redmond, USA).

### 2.2. Construction, Validation, and Clinical Utility of a Nomogram

Patients from the SEER database for 2010–2016 are taken as the training cohort (*n* = 929), and patients from multicenter dataset are taken as the validation cohort (*n* = 51).

We compared clinicopathological characteristics of the training cohort and the validation cohort using the chi-square test. We assessed variables that predicted L.M. in E.S. patients by univariate logistic regression analysis. Subsequently, multivariate logistic regression analysis was used to evaluate each variable at a 0.05 significance level, and the independent factors associated with L.M. were obtained. Based on the multivariable logistic regression analysis, a nomogram has been constructed in the training set. We plotted the receiver operating characteristic (ROC) curves and calculated the area under ROC (AUC) to evaluate the prediction accuracy of the nomogram. The relationship between actual probability and the predicted probability is verified by calibration curves. Moreover, decision curve analysis (DCA) was used to evaluate the clinical utility and value of the nomogram.

The article "Development and Validation of a Novel Clinical Prediction Model to Predict the Risk of Lung Metastasis from Ewing Sarcoma for Medical Human-Computer Interface" was published in 2022. Journal: Comput Intell Neurosci.

## 3. Statistical Analysis

Continuous and categorical variables are expressed as mean ± SD and frequency in this study. All statistical methods, including the *T*-test, chi-square test, Kaplan–Meier analysis, and logistic regression analysis, were conducted via SPSS Statistics software (version 26.0, SPSS Inc., Chicago, USA). *R* software (version 4.0.5, *P* value < 0.05) was applied to complete the nomogram, receiver operating characteristic (ROC) curves, calibration plots, and DCA curves with statistical significance. The results with a significance level less than 0.05 were considered statistically significant, and 95% confidence intervals (CIs) were applied for all analysis.

## 4. Results

### 4.1. Demographic Baseline Characteristics

A cohort of a total of 980 patients was enrolled in this study. Of these, 929 patients from the SEER dataset were assigned to the training cohort and 51 patients from multiple centers were assigned to the validation cohort. Results of the *T*-test and the chi-square test indicated that there was no statistically significant difference between training and validation groups in L.M., age, survival time, sex, primary site, laterality, N stage, surgery, chemotherapy, and bone metastasis at 0.05 significance level (Table 1, *P* > 0.05), but there was significant difference in race, radiation, and *T* stage (Table 1, *P* < 0.05). Afterward, as identified in Table 2, among the total 980 patients, 185 (18.9%) had L.M. and 795 (81.1%) did not have L.M. There is a significant difference of L.M. group and NO-L.M. group in survival time, *T* stage, N stage and *M* stage, surgery, and bone metastasis at 0.05 significance level.

### 4.2. Univariate and Multivariable Logistic Regression Results

There were six significant factors (survival time, N stage, *T* stage, *M* stage, surgery, and bone metastasis) identified by the univariate logistic regression analysis in Table 3. Multivariate logistic regression analysis was further performed, and it showed that *T* stage (T2, OR = 2.545, 95% CI = 1.573–4.117, *P* < 0.001; T3, OR = 3.615, 95% CI = 1.503–8.696, *P* < 0.01; Tx, OR = 2.988, 95% CI = 1.675–5.332, *P* < 0.001), N stage (N1, OR = 4.953, 95% CI = 2.893–8.480, *P* < 0.001), and bone metastasis (yes, OR = 1.887, 95% CI = 1.205–2.954, *P* < 0.01) were independent risk factors, and survival time (OR = 0.988, 95% CI = 0.979–0.997, *P* < 0.01) and surgery (yes, OR = 0.434, 95% CI = 0.294–0.643, *P* < 0.001) were independent protective factors for L.M. in patients with E.S.

The article "Development and Validation of a Novel Clinical Prediction Model to Predict the Risk of Lung Metastasis from Ewing Sarcoma for Medical Human-Computer Interface" was published in 2022. Journal: Comput Intell Neurosci.

For predicting L.M. in patients with E.S., a nomogram was established based on the results of univariate and multivariable logistic regression in the training set (Figure 1(a)). Meanwhile, we designed a medical human-computer interface—an online web calculator (https://drliwenle.shinyapps.io/LMESapp/)—to evaluate the risk of L.M. for each patient. We found that the N stage had the greatest impact on L.M., and surgery had the smallest impact (Figure 1(a)). The AUC in internal validation and external validation was 0.769 (95% CI: 0.740 to 0.795) and 0.841 (95% CI: 0.712 to 0.929), respectively, indicating that the nomogram has a good discriminative ability to assess the status of L.M. (Figures 1(b) and 1(c)). The calibration curve of the nomogram revealed good consistency in training and validation cohorts (Figures 2(a) and 2(b)). The results of the training and validation cohorts consistently showed that the prediction ability of the nomogram was higher than that of a single factor (Figures 2(a) and 2(b)).

The results of validation set suggested that the new model had significantly improved accuracy and reliability for cancer prediction compared with the single factor as shown in Table 4.

### 4.3. Clinical Utility of the Nomogram

The Kaplan–Meier survival curves of the overall survival (O.S.) of the total 980 patients were plotted (Figure 3). The results unveiled that compared with the NO-L.M. group, the survival level of E.S. patients with L.M. significantly decreased much more (*P* < 0.0001).

Meanwhile, we observed that the model had good clinical utility in predicting lung metastasis in both the training and the validation cohorts in E.S. patients. The net benefit of the training cohort was slightly higher than that of the validating cohort, which might be caused due to the limitation of the scale of the validation cohort (Figures 4(a) and 4(b)).

## 5. Discussion

Ewing sarcoma (E.S.) is a rare high-cell malignant round-cell tumor of bone, which occasionally occurs in soft tissue and extra-bone tissue. E.S. is characterized by dissemination and micro-metastasis that cannot be detected by clinical imaging such as CT, PET-CT, or MRI [30]. The most common metastatic site is the lung, followed by distant bone [14]. Previous researchers [10, 12, 14, 15, 17, 20, 21, 35–37] constructed and validated nomograms to predict metastasis and the overall survival and cancer-specific survival in patients with E.S. However, it is innovative to establish a nomogram model combined with data from the SEER database and four independent medical centers to estimate the risk of key predictors of L.M. in E.S. Moreover, we designed a medical human-computer interface (web calculator) as a practical tool for clinicians, using ML algorithm to predict the risk outcomes of patients. ML has the advantage of being highly capable, objective, and repeatable in processing large datasets and reliable data [38–41]. This artificial intelligence-based strategy can be exploited by clinicians to help them select more rational treatment responses [42–45].

The article "Development and Validation of a Novel Clinical Prediction Model to Predict the Risk of Lung Metastasis from Ewing Sarcoma for Medical Human-Computer Interface" was published in 2022. Journal: Comput Intell Neurosci.

In this study, five independent factors (survival time, *T* stage, N stage, surgery, and bone metastasis) were identified associated with L.M. In addition, a nomogram model was built and validated to accurately predict metastasis in patients with E.S.

According to the results of logistic regression, we found that survival time was negatively associated with L.M. as an independent protective factor for the incidence of L.M. in patients with E.S. A study by Leavey et al. indicated that 79% of patients experienced the first recurrence within two years of initial diagnosis. Approximately 30% of them are in the lungs based on 262 cases [46]. Of these independent risk factors for poor prognosis, metastasis appears to be the most common [46], which could cause more death in a short time. It was proved that once the tumor was well controlled and less likely to metastasize, patients would have longer survival.

Furthermore, this paper showed that *T* stage had a negative effect on the occurrence of L.M. in E.S. patients. In Table 3, it is demonstrated that the size of the tumor contributed most to the nomogram, while in1990s, scholars had testified that tumor size is the independent factor for primary metastasis [47], which was similar to subsequent studies [14, 17, 23, 27, 35, 48, 49]. In the aspect of tumor size, Ramkumar et al. proved that tumors with a diameter greater than 118 mm increased the incidence of L.M. by nearly threefold [12]. Ye et al. explained that the 80 mm tumor is prone to have metastasis [13]. The relationship between tumor size and metastasis is worth further study. The rationale behind this can be explained by the fact that large tumors have invaded into surrounding soft tissues, where lymphatics and blood vessels are abundant, promoting the occurrence of lung metastasis [42].In addition, it is difficult to conduct sufficient surgical resection and acquire proper margins [13, 36], which highlights the significance of early detection of E.S. Unfortunately, early diagnosis remains a huge challenge for both patients and doctors as many tumors are painless [50, 51].

Our study indicated that N stage is the most significant predictor for L.M. in patients with E.S. Approximately 30.8% (57/185) of patients with L.M. had N1 and NX status in this study, and the rate of lymph node involvement is 8.2% (80 patients) which is higher than 6.3% in previous studies [52]. According to the results of Table 3, the risk ratios for L.M. in N1 and Nx patients were 4.953 and 1.41, respectively, compared with patients without lymph node metastasis. Because lymphatic vessels are not present in the bone [50], lymph node metastasis and L.M. were more likely to occur when E.S. had invaded into surrounding soft tissues. Given that regional lymph node involvement can be an independent adverse prognostic factor and it is more likely to metastasize [52], FDG-PET scan [53] and even biopsies are recommended for suspected patients with lymph node metastasis.

The article "Development and Validation of a Novel Clinical Prediction Model to Predict the Risk of Lung Metastasis from Ewing Sarcoma for Medical Human-Computer Interface" was published in 2022. Journal: Comput Intell Neurosci.

In addition, the results of logistic regression also revealed that surgery was an independent protective factor. We found that 89% of patients who underwent surgery had no L.M., and only 11% of them had L.M. For patients with E.S., distant metastasis is the main cause of relapse. Modern treatments with more aggressive surgical approaches can prevent distant metastases and improve local control, where the disease-free survival for patients with localized disease may be close to 70% [54, 55]. Surgery was verified to significantly associate with O.S. [15, 32]. It is no doubt that surgery is one of the most successful and vital strategies for the treatment of E.S.

In the present study, patients with bone metastasis had a higher tendency to develop L.M., which was consistent with the statistical results of logistic regression. Approximately 30.8% (57/185) of patients with L.M. had bone metastasis in this study. The most common site of metastasis is the lung, followed by bones [2, 4]. Patients with bone metastasis alone had a worse prognosis than those with L.M. exclusively [3, 4, 13, 56]. Owing to the aggressiveness of extra-pulmonary metastasis, once bone metastasis occurs, it is prone to metastasize to lungs [3, 13, 48]. Therefore, bone metastasis is a key manifestation leading to L.M.

Several limitations of this study should be considered. First, as a retrospective study, potential bias cannot be ignored. Second, a host of factors probably related to L.M. should be included, such as carcinoembryonic antigen (CEA), surgical margin status, detailed plan of radiotherapy and chemotherapy, and vascular invasion. Third, the sample size of external validation was too small.

## 6. Conclusion

We comprehensively assessed the predictors to L.M. in E.S. based on a dataset from the SEER database and four independent medical institutions. A novel nomogram model was constructed to enhance the prediction ability of the risk of L.M. and guide clinicians in individualized precision treatment, which is helpful for follow-up management measures.

The article "Development and Validation of a Novel Clinical Prediction Model to Predict the Risk of Lung Metastasis from Ewing Sarcoma for Medical Human-Computer Interface" was published in 2022. Journal: Comput Intell Neurosci.

## Figures and Tables

**Figure 1:** (a) Nomogram for the risk of pulmonary metastasis for patients with E.S. (b, c) Training cohort and the validation cohort calibration diagrams indicating good consistency.

**Figure 2:** ROC of nomogram for the pulmonary metastasis risk (a) for training group and (b) for validation group.

**Figure 3:** The Kaplan–Meier survival analysis of lung metastasis in patients with E.S.

**Figure 4:** Nomogram decision curve (DCA) for the risk of the lung metastasis. The red curve (number of high risk) indicates the number of people classified as positive (high risk) by nomogram for each threshold probability. The green curve (number of high risk with outcome) represents the number of true positive under each threshold probability. (a) Training group. (b) Validation group.

**Table 1:** Baseline data of the training group and the validation group.

Variable	Level	Overall (*N* = 980)	SEER (training group, *N* = 929)	Multicenter data (validation group, *N* = 51)	*P*
Race (%)	Black	39 (3.98)	39 (4.20)	0 (0.00)	<0.0001
	Others	126 (12.86)	75 (8.07)	51 (100.00)	
	White	815 (83.16)	815 (87.73)	0 (0.00)	
Age (median [IQR])	NA	17.000 [12.000, 27.000]	17.000 [12.000, 27.000]	17.000 [12.500, 30.500]	0.4801
Survival times (median [IQR])	NA	26.000 [11.000, 47.000]	26.000 [11.000, 47.000]	23.000 [12.500, 39.500]	0.8509
Sex (%)	Female	418 (42.65)	395 (42.52)	23 (45.10)	0.828
	Male	562 (57.35)	534 (57.48)	28 (54.90)	
Primary site (%)	Axis bone	431 (43.98)	404 (43.49)	27 (52.94)	0.3936
	Limb bone	317 (32.35)	304 (32.72)	13 (25.49)	
	Others	232 (23.67)	221 (23.79)	11 (21.57)	
Laterality (%)	Left	374 (38.16)	353 (38.00)	21 (41.18)	0.8945
	Not a paired site	296 (30.20)	281 (30.25)	15 (29.41)	
	Right	310 (31.63)	295 (31.75)	15 (29.41)	
T stage (%)	T1	351 (35.82)	331 (35.63)	20 (39.22)	0.0075
	T2	429 (43.78)	404 (43.49)	25 (49.02)	
	T3	39 (3.98)	34 (3.66)	5 (9.80)	
	TX	161 (16.43)	160 (17.22)	1 (1.96)	
N stage (%)	N0	841 (85.82)	797 (85.79)	44 (86.27)	0.3121
	N1	80 (8.16)	74 (7.97)	6 (11.76)	
	NX	59 (6.02)	58 (6.24)	1 (1.96)	
Surgery (%)	No	413 (42.14)	388 (41.77)	25 (49.02)	0.3811
	Yes	567 (57.86)	541 (58.23)	26 (50.98)	
Radiation (%)	No	757 (77.24)	728 (78.36)	29 (56.86)	0.0007
	Yes	223 (22.76)	201 (21.64)	22 (43.14)	
Chemotherapy (%)	No/unknown	58 (5.92)	58 (6.24)	0 (0.00)	0.1248
	Yes	922 (94.08)	871 (93.76)	51 (100.00)	
Bone metastases (%)	No	831 (84.80)	791 (85.15)	40 (78.43)	0.2714
	Yes	149 (15.20)	138 (14.85)	11 (21.57)	
Lung metastases (%)	No	795 (81.12)	754 (81.16)	41 (80.39)	1
	Yes	185 (18.88)	175 (18.84)	10 (19.61)	

**Table 2:** Baseline data for patients presenting with and without lung metastases.

	Level	Overall (*N* = 980)	No (*N* = 795)	Yes (*N* = 185)	*p*
Category (%)	Multicenter data (validation group)	51 (5.2)	41 (5.2)	10 (5.4)	1
	SEER (training group)	929 (94.8)	754 (94.8)	175 (94.6)	
Race (%)	Black	39 (4.0)	27 (3.4)	12 (6.5)	0.133
	Others	126 (12.9)	105 (13.2)	21 (11.4)	
	White	815 (83.2)	663 (83.4)	152 (82.2)	
times (mean (SD))	NA	30.56 (22.65)	32.27 (22.77)	23.22 (20.60)	<0.001
Age (mean (SD))	NA	22.39 (16.45)	22.38 (16.61)	22.43 (15.81)	0.968
Sex (%)	Female	418 (42.7)	347 (43.6)	71 (38.4)	0.221
	Male	562 (57.3)	448 (56.4)	114 (61.6)	
Primary site (%)	Axis bone	431 (44.0)	337 (42.4)	94 (50.8)	0.11
	Limb bone	317 (32.3)	263 (33.1)	54 (29.2)	
	Others	232 (23.7)	195 (24.5)	37 (20.0)	
Laterality (%)	Left	374 (38.2)	306 (38.5)	68 (36.8)	0.734
	Not a paired site	296 (30.2)	242 (30.4)	54 (29.2)	
	Right	310 (31.6)	247 (31.1)	63 (34.1)	
T stage (%)	T1	351 (35.8)	323 (40.6)	28 (15.1)	<0.001
	T2	429 (43.8)	330 (41.5)	99 (53.5)	
	T3	39 (4.0)	23 (2.9)	16 (8.6)	
	TX	161 (16.4)	119 (15.0)	42 (22.7)	
N stage (%)	N0	841 (85.8)	713 (89.7)	128 (69.2)	<0.001
	N1	80 (8.2)	40 (5.0)	40 (21.6)	
	NX	59 (6.0)	42 (5.3)	17 (9.2)	
M stage (%)	M0	662 (67.6)	662 (83.3)	0 (0.0)	<0.001
	M1	318 (32.4)	133 (16.7)	185 (100.0)	
Surgery (%)	No	413 (42.1)	291 (36.6)	122 (65.9)	<0.001
	Yes	567 (57.9)	504 (63.4)	63 (34.1)	
Radiation (%)	No	757 (77.2)	620 (78.0)	137 (74.1)	0.293
	Yes	223 (22.8)	175 (22.0)	48 (25.9)	
Chemotherapy (%)	No/unknown	58 (5.9)	45 (5.7)	13 (7.0)	0.592
	Yes	922 (94.1)	750 (94.3)	172 (93.0)	
Bone metastases (%)	No	831 (84.8)	703 (88.4)	128 (69.2)	<0.001
	Yes	149 (15.2)	92 (11.6)	57 (30.8)	

The article "Development and Validation of a Novel Clinical Prediction Model to Predict the Risk of Lung Metastasis from Ewing Sarcoma for Medical Human-Computer Interface" was published in 2022. Journal: Comput Intell Neurosci.

**Table 3:** Univariate and multifactorial logistic regression analysis of risk factors for lung metastasis in patients with Ewing's sarcoma.

Variables	Univariate OR (95% CI)	*P* value	Multivariate OR (95% CI)	*P* value
Age（years）	1.003 (0.993–1.013)	0.569	—	—
Survival time (months)	0.979 (0.971–0.988)	<0.001	0.988 (0.979–0.997)	<0.01
Race				
White	Ref	Ref	Ref	Ref
Black	1.939 (0.960–3.914)	0.065	—	—
Others	0.750 (0.396–1.456)	0.395	—	—
Sex				
Male	Ref	Ref	Ref	Ref
Female	0.782 (0.558–1.097)	0.154	—	—
Primary site				
Limb bones	Ref	Ref	Ref	Ref
Axis of a bone	1.381 (0.942–2.025)	0.098	—	—
Others	0.965 (0.605–1.540)	0.882	—	—
Laterality				
Left	Ref	Ref	Ref	Ref
Right	1.087 (0.735–1.607)	0.676	—	—
Others	0.941 (0.627–1.413)	0.770	—	—
T stage				
T1	Ref	Ref	Ref	Ref
T2	3.320 (2.102–5.244)	<0.001	2.545 (1.573–4.117)	<0.001
T3	7.881 (3.583–17.336)	<0.001	3.615 (1.503–8.696)	<0.01
TX	4.008 (2.363–6.796)	<0.001	2.988 (1.675–5.332)	<0.001
N stage				
N0	Ref	Ref	Ref	Ref
N1	5.587 (3.405–9.166)	<0.001	4.953 (2.893–8.480)	<0.001
NX	2.316 (1274–4.211)	<0.01	1.410 (0.728–2.733)	0.309
Surgery				
No	Ref	Ref	Ref	Ref
Yes	0.278 (0.196–0.394)	<0.001	0.434 (0.294–0.643)	<0.001
Radiation				
No	Ref	Ref	Ref	Ref
Yes	1.091 (0.736–1.617)	0.663	—	—
Chemotherapy				
No	Ref	Ref	Ref	Ref
Yes	0.791 (0.417–1.500)	0.473	—	—
Bone metastases				
No	Ref	Ref	Ref	Ref
Yes	3.857 (2.607–5.706)	<0.001	1.887 (1.205–2.954)	<0.01

The article "Development and Validation of a Novel Clinical Prediction Model to Predict the Risk of Lung Metastasis from Ewing Sarcoma for Medical Human-Computer Interface" was published in 2022. Journal: Comput Intell Neurosci.

**Table 4:** AUC of the training group and validation group.

Variable	SEER data (training group)			Multicenter data (validation group)		
	AUC	SE	95% CI	AUC	SE	95% CI
Bone metastases	0.606	0.0186	0.573 to 0.637	0.572	0.0604	0.426 to 0.710
N stage	0.599	0.0182	0.567 to 0.631	0.598	0.0787	0.451 to 0.732
Surgery	0.655	0.0199	0.623 to 0.685	0.506	0.0922	0.362 to 0.649
Survival time	0.627	0.0232	0.595 to 0.658	0.544	0.108	0.398 to 0.684
T stage	0.639	0.0201	0.608 to 0.670	0.689	0.0751	0.544 to 0.811
Nomogram	0.769	0.0198	0.740 to 0.795	0.841	0.0634	0.712 to 0.929

## Data Availability

The data used to support the findings of this study are available from the corresponding author upon request.
